The article "Development and psychometric evaluation of the Employee's Workplace Cyberloafing Scale (EWCS)" was published in 2024. Journal: Heliyon.

# Development and psychometric evaluation of the Employee's Workplace Cyberloafing Scale (EWCS)

**DOI:** 10.1016/j.heliyon.2024.e39376

**Published:** 2024-10-15

**Authors:** Harlina Nurtjahjanti, Rahmat Hidayat, Indrayanti Indrayanti

**Affiliations:** a Faculty of Psychology, Universitas Gadjah Mada, Special Region of Yogyakarta, Indonesia; b Faculty of Psychology, Universitas Diponegoro, Semarang, Indonesia

**Keywords:** Employee, Cyberloafing, Psychometric evaluation, Employee's workplace Cyberloafing Scale

## Abstract

Cyberloafing refers to the practice of employees using the Internet for non-work-related purposes during working hours. This study aims to develop a measurement scale for cyberloafing among employees, specifically those working in Indonesia. The research was conducted in two stages. In the first stage, items were developed through a literature review, theme selection using qualitative research, expert review, and item readability testing. The results from this stage were then used in the second stage, which involved psychometric testing of the instruments using Exploratory Factor Analysis (EFA) and Confirmatory Factor Analysis (CFA). A total of 726 administrative employees from seven state universities in a major city on Java Island, Indonesia, participated in the study. The EFA test, conducted on 300 respondents, revealed a four-factor structure consistent with the construct. Subsequently, CFA was performed on 426 respondents, confirming the model's adequacy with four factors: entertainment, interaction, transaction, and recreation. The EFA results, validated by the CFA test, indicated that these factors accounted for 45.98 % of entertainment, 9.40 % of interaction, 6.36 % of transactions, and 5.15 % of recreation in cyberloafing behavior. The findings demonstrate that the Employee Workplace Cyberloafing Scale (EWCS) is a valid and reliable instrument for assessing cyberloafing among Indonesian workers. The EWCS serves as a versatile tool for both government and private sectors, providing critical insights into personal internet usage during work hours. Beyond mere monitoring, it reveals patterns indicative of addictive online behavior, empowering organizations to develop tailored intervention programs that address and mitigate employee mental health challenges.

## 1 Introduction

Internet technology allows individuals to exist in two spaces simultaneously: actual space and virtual space. For instance, while working at a desk (actual space), an employee can chat with friends in another city via social media (virtual space) or watch the World Cup live through streaming channels (virtual space). This duality of existence can lead to various issues, such as cyberloafing. Cyberloafing is defined as using company internet access for non-work-related activities during working hours [1]. The increased popularity of personal technology, including computers, tablets, and smartphones, all connected to the internet, has made cyberloafing feasible [2]. It is nearly impossible to monitor and restrict the use of personal devices that are connected to work devices [3]. This blurs the line between work-related activities and non-work-related interests. As a result, there is a growing trend of employees using the Internet for personal purposes during work hours [4].

The article "Development and psychometric evaluation of the Employee's Workplace Cyberloafing Scale (EWCS)" was published in 2024. Journal: Heliyon.

For companies, cyberloafing can lead to significant losses, such as increased vulnerability to cyber attacks and financial losses due to higher internet costs and decreased worker productivity. Employees addicted to negative content, such as adult sites and online gambling, can underperform, resulting in poor company performance. Consequently, the phenomenon of cyberloafing among workers has garnered attention in academic research. Weissenfeld et al. (2019) [5] conducted a literature review, identifying 145 articles on cyberloafing published from 2003 to 2017. Similarly, Tandon et al. (2021) [6] identified 87 articles from 2001 to 2021. Most of these studies were conducted in developed countries, including the United States, United Kingdom, South Korea, and Singapore. Field research has also shown that workers engage in cyberloafing for various reasons, including economic benefits from online buying and selling activities [7], social media use for conversation and entertainment [8], and accessing adult and online gambling sites [9].

The widespread phenomenon of cyberloafing among company workers has prompted research aimed at reducing this behavior. Efforts include developing strict and effective company control mechanisms that are applied fairly to all employees [10]. Additionally, understanding cyberloafing can help redirect employees towards positive activities, such as reading news or interacting with family and friends. These positive interactions can foster stable and positive emotions, thereby encouraging greater productivity at work [11].

Even though cyberloafing behaviour has a few positive aspects, it primarily has negative impacts on both employees and the organization as a whole. Therefore, instruments for measuring cyberloafing and its consequences on employee mental health in the workplace are needed. In this regard, some researchers have developed cyberloafing scales [e.g., Refs. [2,12]. Lim's (2002) [12] scale, which includes only two components—browsing activities and email—is one of the most widely used instruments in cyberloafing research. Considering the tremendous development in internet technology in recent years, some authors suggest that this instrument is outdated [7]. Additionally, these instruments may include statements that are considered taboo or not yet familiar and entrenched in the Indonesian work environment, such as investment sites, adult-oriented websites, and personal email use. Overall, existing scales are no longer relevant for measuring employee cyberloafing within a contemporary framework. This research aims to address this urgency by developing a psychometric evaluation scale specifically designed to measure cyberloafing behavior among employees working in Indonesia.

The article "Development and psychometric evaluation of the Employee's Workplace Cyberloafing Scale (EWCS)" was published in 2024. Journal: Heliyon.

## 2 Literature review

### 2.1 Cyberloafing

Etymologically, cyberloafing comes from the words “cyber” and “loafing” [13]. Cyberloafing is a common work-related behavior where employees use technology for personal gain rather than work-related tasks [14,15]. This phenomenon is widely recognized as a form of counterproductive work behavior, with the potential to lead to misuse, theft, and sale of confidential data or sensitive information within an organization's information technology system. Other terms frequently used to describe this behavior include cyberslacking [16,17], personal internet usage [15,18], internet addiction [17,19], and cyber-deviance [18]. Cyberloafing has been extensively studied as a mediating mechanism linking negative events in the workplace to employee behavioral responses [19,20].

The forms of cyberloafing behavior are varied, with the most common being sending and receiving electronic messages for personal interests [[20], [21], [22]], browsing websites, visiting entertainment sites, and making online purchases [23]. The phenomenon of visiting and surfing on social networking sites is also widely observed [4,24]. Many studies have been conducted on the impact of cyberloafing, particularly for organizations. Conceptually, this impact is closely related to counterproductive withdrawal behavior [25,26]. This activity engrosses employees in personal internet use during working hours, resulting in divided attention and limiting their ability to fully focus on their work. Another study reported that employee involvement in cyberloafing can drain mental resources, thereby reducing the level of employee engagement in the workplace [27]. Additionally, engagement in cyberloafing at work is exacerbated by the tendency for addictive behavior in technology use outside of work life [28].

Some research has highlighted the positive benefits of cyberloafing. This perspective is based on the fact that today's employees increasingly work long hours, making them vulnerable to stress and fatigue [29]. Kim et al.'s (2016) [30] research found that employees' use of social media for non-work purposes at work can offer a respite, allowing them to recover mental and cognitive resources, which in turn contributes to improvements in subsequent work behavior [31]. Recent meta-analytic findings suggested that employees engage in cyberloafing in response to increases in their workload [32]. The contradictory results in cyberloafing-related research are not particularly surprising, given the inconsistent use of terminology in this domain, leading to uncertainty regarding the appropriate approach to measuring cyberloafing.

The article "Development and psychometric evaluation of the Employee's Workplace Cyberloafing Scale (EWCS)" was published in 2024. Journal: Heliyon.

### 2.2 Cyberloafing scale development

In the last two decades, several researchers have conducted research on the development of cyberloafing instruments. Lim (2002) [12] developed a cyberloafing scale consisting of 11 items covering two factors, namely browsing activities and e-mailing activities. This scale is a measuring tool that is widely used as a reference in subsequent scale developments. Furthermore, Lim & Teo (2005) [33] developed the cyberloafing scale from Lim (2002) into 13 items to examine the prevalence and seriousness of various cyberloafing activities. Meanwhile, Blau et al. (2006) [34] built a new instrument by conducting a survey using 16 items, of which 10 items were adopted directly from Lim's (2002) [12] scale. Three forms of cyberloafing that have been measured are non-work-related e-mail cyberloafing, browsing-related cyberloafing, and interactive cyberloafing.

In its development, Blanchard & Henle (2008) [35] conducted exploratory research using a scale developed by Lim (2002) [12] consisting of 21 items, and distinguished two forms of cyberloafing, namely serious cyberloafing and minor cyberloafing. Furthermore, Askew et al. (2014) [36] conducted additional research to investigate the topic in more depth using 19 questions, which was an extension of the cyberloafing scale developed by Lim (2002) [12]. The study found a multidimensional construct of cyberloafing in a 12-item cyberloafing scale and produced four components, namely social, informational, leisure, and virtual-emotional activity. Furthermore, Yildiz and Örücü (2014) [37] used 19 questions to measure cyberloafing, including 8 questions derived from Lim's (2002) [12] scale, 4 questions adopted from Blanchard & Henle's (2008) [35] scale, as well as 7 additional questions aimed at collecting demographic information. Meanwhile, the latest research by Zhong et al. (2022) [38] has developed an instrument to evaluate employee engagement in the use of online resources to search for news and information related to COVID-19 during working hours. The instrument consists of six items developed based on the scale from Lim & Teo (2005) [33] and constructed based on available literature.

The article "Development and psychometric evaluation of the Employee's Workplace Cyberloafing Scale (EWCS)" was published in 2024. Journal: Heliyon.

Of all the cyberloafing instruments that have been developed by academics, two weaknesses need to be corrected. First, the existing measuring instruments use a limited number of items, so they are unable to adequately represent cyberloafing as a multidimensional phenomenon. Organizational behavior research increasingly uses multidimensional constructs to link predictors to more comprehensive outcomes [39,40]. Cheung et al. (2023) [41] added that measuring the complexity of a phenomenon requires a multidimensional instrument so it requires a greater number of items in the measurement model compared to a single-dimensional construct [42]. Second, the use of questionnaires to obtain data which is then used as a basis for compiling items, has the potential to cause bias in the results because the effectiveness of the questionnaire depends on the researcher's understanding of the factors that influence participant responses [43].

Table 1 above presents previous research findings on cyberloafing activities based on the types of sites employees browse. The types of sites have increased over the years. For example, Lim (2002) found that employees visited news, sports, entertainment, investment, non-job-related, online shopping, and adult-oriented sites. Lim and Teo (2005) also included online gameplay sites in their research, while Bali et al. (2006) added sites related to additional income at work. Lastly, Blanchard and Henle (2008) concluded that employees visited news, sports, stock, financial, gambling, virtual communities, adult-oriented, online shops, online auctions, personal websites, blogs, and music sites. Employees also use the office internet for non-work-related communications, such as checking, receiving, sending, and using email chat for non-work purposes.

**Table 1:** Exploratory factor analysis of cyberloafing items.

Researchers	Cyberloafing Items	
	Browsing Activities	Email Activities
Lim (2002) [12]	● General news sites. ● Sports related websites. ● Entertainment related websites. ● Investment related websites. ● Non-job related websites. ● Download non-work related information. ● Shop online for personal goods. ● Adult-oriented (Sexually explicit) websites.	● Check non-work related email. ● Receive non-work related email. ● Send non-work related email.

Lim & Teo (2005) [33]	● General news sites. ● Sports related websites. ● Entertainment related websites. ● Investment related websites. ● Non-job related websites. ● Download non-work related information. ● Shop online for personal goods. ● Adult-oriented (Sexually explicit) websites. ● Play online games.	● Check non-work related email. ● Receive non-work related email. ● Send non-work related email. ● Instant messaging/chat online (IRC).
Blau et al. (2006) [34]	● General news sites. ● Sports related websites. ● Entertainment related websites. ● Investment related websites. ● Non-job related websites. ● Download non-work related information. ● Shop online for personal goods. ● Download online games. ● Play online games. ● Use the internet to gain additional income while at work.	● Check non-work related email. ● Receive non-work related email. ● Send non-work related email. ● Post messages on non-work related items. ● Chat with other people in online chat rooms. ● Chat with other people with instant messenger.

Blanchard & Henle (2008)	● Visit news sites. ● Visit sports sites. ● Visit stock sites. ● Visit financial sites. ● Visit gambling sites. ● Visit virtual communities. ● Visit adult-oriented sites. ● Shop online. ● Online auctions. ● Maintain personal web page. ● Check personals. ● Read blogs. ● Download music.	● Check non-work related email. ● Receive non-work related email. ● Send non-work related email. ● Participate in chat rooms.

To further explore cyberloafing in Indonesia, a study was conducted with 28 participants to inquire about the sites they visit during work and how they use the internet for office communication (see Table 2). Surprisingly, the study found that employees in Indonesia visit various sites, including those for personal information, entertainment (e.g., online video viewing, gaming, and music), financial transactions, learning, business, and self-expression (e.g., TikTok, YouTube, and Instagram). Regarding internet use for communication, the preliminary study revealed that participants used the internet for personal emails, social media chats and video calls, posting updates on social media, commenting, liking, and sharing photos, videos, and articles while at work.

The article "Development and psychometric evaluation of the Employee's Workplace Cyberloafing Scale (EWCS)" was published in 2024. Journal: Heliyon.

**Table 2:** Exploratory Factor Analysis of EWCS Items (Source: authors).

Browsing Activities	Email Activities
● Shopping online and e-commerce activities to fulfil personal requirements. ● Accessing digital banking for personal transactions. ● Playing online game. ● Watching entertainment shows from YouTube, TikTok, Instagram, online TV, and others. ● Listening to music online. ● Reading online news portals to search for up-to-date information that is not work-related. ● Updating social media status for entertainment (WhatsApp, tweets or Insta stories). ● Downloading online entertainment apps. ● Watching online videos via vlogs, online tutorials, online learning, webinars, or others to improve personal competence. ● Downloading digital learning applications to increase personal capacity, which is unrelated to work. ● Building business opportunities as a blogger, YouTuber, design service, online shop owner, content creator or others. ● Creating creative non-work-related video content on YouTube, TikTok, Instagram or other platforms.	● Replying to messages unrelated to work through personal chat, direct messages, voice notes, personal emails, or other things. ● Sending messages using personal chat, direct messages, voice notes, personal emails or other things that are not related to work. ● Using the telephone features of WhatsApp, Facebook Messenger, Skype, or others to communicate outside work matters. ● Responding to others' post by commenting, liking, follow-unfollowing account or other activities. ● Sharing photos, videos, articles, websites, or others to express oneself in the middle of work-related activities.

Most of the cyberloafing items in the instrument we developed adopted several previous researchers, namely cyberloafing for information, entertainment, sports and economic motives. However, we excluded certain item because, as previously discussed, these activities are often kept confidential by the employees involved and are not typically shared with others. Apart from that, most of the cyberloafing items that we develop are related to entertainment because the majority of workers in Indonesia need entertainment and relaxation for a moment from work fatigue or to avoid pressure and stress due to work or economic related items in the form of developing business opportunities, especially digital-based ones, increase income or access financial institutions to obtain loans and capital. We also include several items from the positive perspective of cyberloafing such as accessing news or online articles to broaden insight and increase knowledge.

## 3 Method

This research is a cross-sectional study employing an online survey questionnaire distributed to state university (PTN) employees. Before data collection, a prior consent form was submitted to all participants to be part of the research. In the context of data management, information obtained from participants is stored in an anonymous form to ensure that the data cannot be linked to any information to identify research participants. The sampling procedure used in this research involved the use of judgment sampling. The inclusion criteria for this study included several considerations, including at least two years of work experience, using the internet for work, and having at least one social media application/account, such as WhatsApp, Facebook, and Instagram. All EWCS items are scored using a 5-point Likert scale of (1) “Never”, (2) “Rarely”, (3) “Sometimes”, (4) “Often”, and (5) “Always".

The article "Development and psychometric evaluation of the Employee's Workplace Cyberloafing Scale (EWCS)" was published in 2024. Journal: Heliyon.

### 3.1 Procedure (initial scale construction)

Development and validation of the Employee's Workplace Cyberloafing Scale (EWCS) utilized construction parameters from Hinkin (1995) [44] and DeVellis (2017) [45]. This parameter includes four stages as depicted in Fig. 1: 1) theoretical investigation, 2) qualitative inquiry, 3) item generation, and 4) psychometric evaluation.

**Fig. 1:** The Employee's Workplace Cyberloafing Scale (EWCS) development process.

Fig. 1 outlines the research procedure, which comprises four distinct phases. Phase 1 begins with a comprehensive theoretical assessment, encompassing an extensive literature review and establishing a conceptual definition. Moving to Phase 2, qualitative inquiry takes precedence, involving implementing semi-structured interviews and identifying overarching themes and sub-themes. Phase 3 emphasizes item generation, where intricate items are meticulously crafted, subjected to expert scrutiny, and eventually culminate in developing a final draft questionnaire. Finally, Phase 4 underscores psychometric evaluation, which encompasses both exploratory factor analysis (EFA) and confirmatory factor analysis (CFA) to assess the research instrument's underlying structural framework and validity.

A total of 20 initial EWCS items were created using inductive and deductive methods. The deductive method for establishing a conceptual definition of cyberloafing was carried out using a mini-systematic literature review [46]. Literature studies are very important in understanding the phenomenon being studied, as well as building a theoretical framework for quantitative research construction [47,48]. To refine the parameters of the measurement construct and ensure its coverage, this research used an inductive method utilizing a qualitative phenomenological approach. Qualitative phenomenology methodology allows researchers to understand the meaning of individuals' lived experiences of a phenomenon [49,55]. The process of converting qualitative data into quantitative data to construct the items in this study followed Sandelowski's contingent design guidelines which involve coding data during the data analysis process [[50], [51], [52]]. Phase 1 and Phase 2 of these studies produced the main components of EWCS, including the need for entertainment, interaction, information, transactions, and skills.

After preparing the items, an internal evaluation was then carried out by involving expert participation to analyze the relevance of each item according to the concept. The evaluation assessment was carried out by 17 experts who met certain criteria, such as having active experience in instrument development research, active involvement in the field of psychological research, and/or demonstrating competence in the field of psychometrics. The results of the validity test using Aiken's V coefficient [53] showed that all items in the EWCS were considered valid, with validation values ranging from 0.73 to 0.98. Specifically, 17 instrument items were found to have an Aiken index above 0.81. The item with the lowest value (0.78) is “Listening to music online”, while the items with the highest value (0.98) include: “Sharing photos, videos, articles, websites, or others to express oneself in the middle of work-related activities”, “Responding to others' post by commenting, liking, follow-unfollowing account or other activities”, and “Sending messages using personal chat, direct messages, voice notes, personal emails or other things that are not related to work.” Based on the results of this expert study, we reviewed several instrument items with a focus on the editorial aspects of the statement. After a discussion process between the research team members, 20 items were agreed upon for further testing. Next, the EWCS was tested on three participants (n = 3) to confirm the face validity. No changes were made to the items according to the feedback provided by participants. Of the initial 20 items, all items with five components were successfully retained for further testing.

The article "Development and psychometric evaluation of the Employee's Workplace Cyberloafing Scale (EWCS)" was published in 2024. Journal: Heliyon.

### 3.2 Population and sample

The research sample of this research was from several administrative employees recruited from seven state universities in Semarang, Central Java, Indonesia. Of the 749 survey data entered, 23 data were excluded because they did not match the predetermined sample criteria, resulting in a response rate of 96 %. A total of 726 valid data were then used for analysis purposes referring to the opinions of Kline (2011) [54].

Based on Byrne's (2011) [55] recommendation, to reduce the significant impact of certain sample results on the reliability and validity of the research, participants were divided into two sub-samples randomly. Then, we performed a series of Chi-square tests to assess whether there were statistically significant differences in the proportions of characteristics between sample A (EFA testing) and sample B (CFA testing). Based on the results obtained, there were no significant differences in the characteristics of the two samples based on gender, age, education, employee status, length of service, and position, namely gender χ2 (1, N1 = 300, N2 = 426) = 0.079, p = 0.801; age χ2 (3, N1 = 300, N2 = 426) = 1.000, p = 0.778; education level χ2 (4, N1 = 300, N2 = 426) = 2.367, p = 0.669; employee status χ2 (3, N1 = 300, N2 = 426) = 0.187, p = 0.980; position χ2 (1, N1 = 300, N2 = 426) = 0.131, p = 0.717; tenure χ2 (3, N1 = 300, N2 = 426) = 1.064, p = 0.786.

The article "Development and psychometric evaluation of the Employee's Workplace Cyberloafing Scale (EWCS)" was published in 2024. Journal: Heliyon.

The number of respondents was 726 people who were valid and then divided into two groups, namely sample A for the Exploratory Factor Analysis (EFA) analysis of 300 people and sample B for the Confirmatory Factor Analysis (CFA) analysis of 426 so that it could be ensured that no respondents were involved in both analyses. We used 300 data to perform EFA. At this testing stage, sample A consisted of 144 women (48.0 %) and 156 men (52.0 %), whose mean age was 38.9 years (SD = 9.04). A total of 50.3 % of participants had a bachelor's degree level of education; 44.30 % were civil servants, 92.0 % had staff positions, and 129 participants had a working period of between 11 and 20 years (43.0 %). In the CFA stage, data from sample B of 426 were used. Participants consisted of 209 women (49.1 %) and 217 men (50.9 %), whose average age was 38.72 years (SD = 8.68). A total of 46.0 % had a bachelor's degree level of education, and 43.7 % were civil servants. A total of 184 participants had a working period of between 11 and 20 years (43.2 %), and 7.3 % of participants were leaders.

### 3.3 Data analysis

EFA was carried out to confirm the factor structure in the form of a 20-item scale analyzed using SPSS 26 software. The suitability of the factor structure was based on the results of the EFA with the data assessed using Confirmatory Factor Analysis (CFA) carried out with Mplus 8.3.

## 4 Results and discussion

### 4.1 Exploratory factor analysis (EFA)

EFA was used to analyze the main constructs of the EWCS instrument and test its internal reliability. Before conducting EFA, the results of the item reduction analysis were confirmed. Evaluation of the psychometric properties of the EWCS was carried out using several reliability testing methods. First, univariate normality was determined by examining the distribution of kurtosis and skewness on each observed variable. Data are considered normal if skewness is between −2 and +2 and kurtosis is between −7 and +7 [55]. Second, the item-total correlation technique was used to avoid redundancy and multicollinearity. This was done to identify pairs of items that were too highly correlated (r > 0.80). Next, the Pearson correlation coefficient was used to measure the relationship between variables, and the r-coefficient values ranged from 0.70 to 1.00 indicating the existence of a strong correlation. Third, the consistency of the items was tested. Adriana Taveira et al. (2024) [56] proposed that item-total correlations with scores **>** 0.30 indicate acceptable item discrimination. Meanwhile, to measure the internal consistency of the EWCS, Cronbach's alpha technique was used, where high reliability is indicated by an alpha value > 0.80.

The article "Development and psychometric evaluation of the Employee's Workplace Cyberloafing Scale (EWCS)" was published in 2024. Journal: Heliyon.

Table 3 shows that the lowest average score is 2.263 with SD = 1.194, and the highest average score is 3.110 with SD = 1.184. The mean total score was 55.033 with SD = 14.797. The lowest skewness value was 0.077, and the highest skewness value was 0.714. The lowest kurtosis value is 1.005, and the highest kurtosis value is 0.165. Meanwhile, the total score produces skewness of 0.692 and kurtosis of 0.695. This means that no outliers have been identified because the items have skewness and kurtosis values outside ± 2, so it can be stated that all items have a normal distribution. Furthermore, the correlation results between variables range from 0.138 to 0.797, indicating a high correlation. Item discrimination testing produced a correlation coefficient ranging from 0.388 to 0.752 and the reliability test produced a Cronbach's alpha value of 0.935. These two findings indicate that all items in the EWCS have strong discrimination abilities and the items correlate well with each other in measuring the same construct. These results also indicate that no items were identified as problematic, and as a result, no items were removed as a result of the analysis.

**Table 3:** Mean, standard deviation, skewness, and kurtosis (N = 300).

Indicator	Mean	Standard deviation	Skewness	Kurtosis
Item 1	2.960	0.991	0.164	−0.358
Item 2	2.487	1.172	0.383	−0.595
Item 3	3.077	0.945	0.372	−0.301
Item 4	3.057	1.015	0.234	−0.566
Item 5	2.263	1.194	0.571	−0.632
Item 6	3.110	1.184	0.077	−1.005
Item 7	2.500	1.049	0.709	0.165
Item 8	3.053	1.078	0.136	−0.825
Item 9	2.690	1.057	0.714	−0.084
Item 10	2.947	1.102	0.287	−0.647
Item 11	2.650	1.125	0.310	−0.591
Item 12	3.030	0.955	0.218	−0.370
Item 13	2.887	1.048	0.264	−0.550
Item 14	2.347	1.106	0.639	−0.120
Item 15	2.830	1.191	0.093	−0.823
Item 16	2.703	1.137	0.190	−0.742
Item 17	2.833	1.165	0.188	−0.745
Item 18	2.780	1.115	0.181	−0.734
Item 19	2.390	1.215	0.399	−0.892
Item 20	2.440	1.251	0.369	−0.939

Total	55.033	14.797	0.692	0.695

Interval consistency = 0.935				

The next step was conducting an assessment of sample adequacy. The results of the research produced a KMO value exceeding 0.9, indicating that the data met the criteria for factor analysis and the p-value was less than 0.05, indicating that there was a significant correlation between variables. Meanwhile, the results of Bartlett's Test of Sphericity show a statistically significant value of less than 0.05, this shows that all items have a significant correlation (see Table 4 based on the findings, it can be concluded that the EWCS consisting of 20 items is considered suitable for factor analysis).

The article "Development and psychometric evaluation of the Employee's Workplace Cyberloafing Scale (EWCS)" was published in 2024. Journal: Heliyon.

**Table 4:** KMO dan Bartlett Test of Sphericity for the Employee's Workplace Cyberloafing Scale (EWCS).

Kaiser-Meyer-Olkin measure of sampling adequacy		0.931
Bartlett's Test of Sphericity	Approximate chi-square adequacy	3762.786
	Df	190
	Sig.	0.000

In the final EWCS model, the analysis results showed that all items had factor loadings above 0.5, so no items were deleted. Among the four factors, there was one factor consisting of two items retained because it did not have a factor loading value below 0.2. A total of 20 items were retained for further analysis. A principal components analysis conducted on the 20 items of the EWCS revealed four components with factor loadings ranging from 0.555 to 0.807. These components can be seen in Table 2. These results were supported by the scree plot providing evidence of the four-factor structure of the EWCS (see Fig. 2).

**Fig. 2:** Scree plot for the factor analysis of the Employee's Workplace Cyberloafing Scale (EWCS) (20 items).

The final step of EFA involved variable evaluation that showed a significant correlation with a particular factor and then assigned a label to that factor. Labeling is highly dependent on the definition provided by the researchers, the theoretical framework used, and the use of inductive reasoning [50]. Conceptually, five dimensions were found in EWCS based on a combination of a literature review approach and a qualitative inquiry, namely entertainment, interaction, information, transactions, and skills. The results of EFA based on eigenvalues produced four factors that corresponded to the construct (see Table 5). The two factors, namely interaction and transaction, were in line with the factors that had previously been created. The entertainment factor gained additional items from the skill and information factors. A new factor was formed, namely, one item came from the entertainment factor and one item came from the skills factor. After examining the item structure, the available literature, and the findings obtained from the qualitative investigation in phases 1 and 2 were referred to ensure the assignment of appropriate labels to the four outcome factors resulting from the EFA analysis. We call these factors the need for entertainment, interaction, transactions, and recreation.

**Table 5:** Items and factor loadings for the Employee's Workplace Cyberloafing Scale (EWCS) (N = 300).

Items	Factor loading value			
	Entertainment	Interaction	Transaction	Recreation
Watching entertainment shows from YouTube, TikTok, Instagram, online TV, and others.	**0.775**	0.295	0.160	0.073
Viewing WhatsApp status updates, tweets or Insta stories for entertainment.	**0.716**	0.109	0.250	0.310
Downloading online entertainment apps that I need.	**0.807**	0.319	0.090	0.092
Listening to music online.	**0.765**	0.282	0.059	0.114
Accessing online news portals to search for up-to-date information that is not work-related/Accessing online news portals to seek current non-work-related information.	**0.608**	0.168	0.521	0.051
Reading online articles unrelated to the work context to broaden the horizons.	**0.595**	0.139	0.442	0.047
Visiting online shopping platforms to look for the latest information regarding product quality, promotions, prices, online customer reviews or others	**0.612**	0.186	0.424	0.073
Watching online videos via vlogs, online tutorials, online learning, webinars, or others to improve personal competence.	**0.568**	0.116	0.249	0.467
Downloading digital learning applications to increase personal capacity, which is unrelated to work.	**0.650**	0.080	0.127	0.444
Building business opportunities as a blogger, YouTuber, design service, online shop owner, content creator or others.	**0.613**	0.092	0.183	0.488
Using the telephone features of WhatsApp, Facebook Messenger, Skype, or others to communicate outside work matters.	0.246	**0.726**	0.341	0.029
Sharing photos, videos, articles, websites, or others to express oneself in the middle of work-related activities.	−0.043	**0.555**	−0.055	0.463
Replying to messages unrelated to work through personal chat, direct messages, voice notes, personal emails, or other things	0.251	**0.784**	0.301	0.094
Responding to others' post by commenting, liking, follow-unfollowing account or other activities.	0.266	**0.719**	0.264	0.150
Sending messages using personal chat, direct messages, voice notes, personal emails or other things that are not related to work.	0.319	**0.763**	0.264	0.057
Engaging in shopping transactions to meet personal needs, such as ordering food, paying bills, purchasing credit/quotas, etc	0.363	0.324	**0.685**	0.093
Accessing digital banking services using internet banking, phone banking or other services for personal transactions.	0.079	0.282	**0.755**	0.230
Engaging in e-commerce activities to fulfil personal requirements	0.226	0.293	**0.743**	0.160
Playing online game	0.351	0.046	0.077	**0.656**
Creating creative non-work related video content on YouTube, TikTok, Instagram or other platforms	0.076	0.150	0.190	**0.752**

Eigenvalues	1.030			

% variance explained	5.151			

Based on PCA, the factors from the retained EWCS explained 66.90 % of the total variance. The first factor (Eigenvalue = 45.98), which explained 45.98 % of the variance, was formed by items measuring the need for entertainment (10 items). The second factor (Eigenvalue = 1.88), explaining 9.40 % of the variance, was formed by items measuring the need for interaction (5 items). The third factor (Eigenvalue = 1.27) explained another 6.36 % of the variance and was the transaction dimension (3 items) formed by items measuring the need for transactions. The fourth factor (Eigenvalue = 1.03) explained 5.15 % of the variance and was the recreation dimension (2 items) formed by items measuring the need for fun.

The article "Development and psychometric evaluation of the Employee's Workplace Cyberloafing Scale (EWCS)" was published in 2024. Journal: Heliyon.

### 4.2 Confirmatory factor analysis (CFA)

Before carrying out CFA, the same steps as the previous stage (EFA) were carried out, namely evaluating the extent of the instrument's psychometric properties using several reliability testing methods. The results of the multivariate normality test showed that the EWCS data was normally distributed. Correlation values between variables ranged from 0.724 to 0.881, indicating no risk of internal consistency. The correlation coefficients of the EWCS items ranged from 0.868 to 0.962, indicating that these items had high discriminatory power. Meanwhile, the reliability test results showed high reliability for all items with reliability coefficient values ranging from 0.918 to 0.975.

All factors including entertainment, interaction, transaction, and recreation were classified to validate the EWCS factor structure of 20 items. In this analysis, the existing data set was tested with a model of four identified factors obtained from EFA. Meanwhile, a one-factor model as an alternative model was proposed to further investigate the validity of the EWCS and determine the most representative data set.

The construct validity of the EWCS and its psychometric performance was evaluated through the application of CFA using an estimation parameter model based on the maximum likelihood estimation method. Model fit assessment utilized several fit indices recommended by Ref. [51] with the following cutoff values: a value lower than 0.08 for the Root-Mean-Squared Error of Approximation (RMSEA), a value of 0.09 or higher for the Comparative Fit Index (CFI) and Tucker–Lewis Index (TLI), a value smaller than 0; p values are greater than 0.05 for Chi-square, and values of 0.08 or lower for Standardized Root Mean Square Residual (SRMR). To determine the criteria for the suitability of the model to the data, we referred to the guidelines provided by Hu and Bentler (1999) [57]. These guidelines recommended the use of at least two indices that meet the cutoff value, such as the RMSEA, CFI, and TLI indexes [58].

In the one-factor model of the EWCS construct, the RMSEA value was 0.129 and the chi-square value was 1376.148 with a probability value = 0.000 indicating an unsatisfactory fit. Meanwhile, the CFI value was 0.893 and the TLI value was 0.881, which was slightly below the criteria, indicating an unsatisfactory match. Meanwhile, the SRMR value of 0.037 indicated a satisfactory match. In general, it can be concluded that the one-factor EWCS model did not show a good fit (poor fit) to the index values.

The article "Development and psychometric evaluation of the Employee's Workplace Cyberloafing Scale (EWCS)" was published in 2024. Journal: Heliyon.

Next, these results were compared with the CFA results on the four-factor model of EWCS constructs (see Table 6). Most of the model fit indices have met the cutoff value suggested by Hu dan Benter (1999) [57]. Fig. 3 showed the RMSEA value of 0.079 indicated an acceptable fit because the value was smaller than 0.08. Meanwhile, the CFI value of 0.961 and the TLI value of 0.955 overall exceeded 0.90, indicating an acceptable fit. Another fit index, an SMSR value of 0.025 indicated a satisfactory fit. Meanwhile, the chi-square value was less than the cutoff value used for goodness of fit, namely 611.538. However, the chi-square test was sensitive to sample size, especially above 400, leading to model rejection in large sample sizes [53,59]. Therefore, the model fit was evaluated using the RMSEA, CFI, TLI, and SRMR indices that met the cutoff points, excluding the chi-square index, as suggested by Ref. [54].

**Table 6:** Fit indices for confirmatory factor model of the one- and four-factor models.

Model	χ2	*P Value*	RMSEA	CFI	TLI	SRMR
One-factor model	1376.148	0.000	0.129	0.893	0.881	0.037
Four-factor model	611.538	0.000	0.079	0.961	0.955	0.025

Notes*. Absolute indexes: χ2 = Chi-square. Relative indexes: CFI* = *Comparative Fit Index; TLI = Tucker–Lewis Index. Fit indexes for comparing non-nested models: RMSEA = Root-Mean-Square Error of Approximation, SRMR* = *Standardized Root Mean Square Residual.*

**Fig. 3:** Four-component CFA model with standardized loading.

### 4.3 Convergent validity

After the multidimensional EWCS was established, the next step was to test the construct validity of the EWCS. This validity was determined using two criteria, namely convergent validity and discriminant validity. Convergent validity consists of factor loadings, average variance extracted (AVE), and composite reliability (CR) as shown in Table 7 below.

**Table 7:** Descriptive statistics and correlations among factors for the Employee's Workplace Cyberloafing Scale (EWCS).

Factor	Ave	Mean	*S.D.*	1	2	3	4
*Entertainment*	0.801	26.857	12.079	**0.975**			
*Interaction*	0.792	13.418	5.744	0.862^a^	**0.950**		
*Transaction*	0.818	7.460	3.718	0.881^a^	0.893^a^	**0.927**	
*Recreation*	0.849	4.697	2.720	0.809^a^	0.734^a^	0.754^a^	**0.918**

*Note*: Values on the diagonal are Cronbach's alpha estimates.

*p* < 0.05 (*one-tailed tests).*

a *p* < 0.01 (*one-tailed tests*).

The article "Development and psychometric evaluation of the Employee's Workplace Cyberloafing Scale (EWCS)" was published in 2024. Journal: Heliyon.

In this study, all factor loadings exceeded 0.8, exceeding the threshold set at 0.7 (Hair et al., 2010). Factor loadings ranged between 0.838 and 0.946. and the AVE of these results was above the minimum threshold of 0.05, with a range between 0.792 and 0.849, confirming the convergent validity of the instrument [56]. The highest AVE was entertainment, namely 0.975, followed by interaction and transactions of 0.950 and 0.927. The lowest AVE was recreation, namely 0.918. Based on the findings presented in Table 7, all AVE and CR values were greater than 0.5, indicating strong evidence of convergent validity for each construct.

Apart from establishing convergent validity, a discriminant validity test was carried out. Discriminant validity was related to the extent to which a construct can be differentiated empirically from other constructs in the model. Discriminant validity was assessed by comparing the AVE value of each construct with the squared correlation between the same construct and all other constructs in the structural model [60]. The results summarized in Table 7 showed that the AVE values for all constructs exceeded the correlation values with other constructs, as determined by the criteria of Fornell and Larcker (1981) [60]. This showed that discriminant validity was also met.

## 5 Discussion

This research aims to develop a valid and reliable instrument to measure cyberloafing in the work context in Indonesia because of the need for a new instrument to evaluate personal internet use among employees [1,25,31] supports international cyberloafing research and its global applications. Developing the Employee's Workplace Cyberloafing Scale (EWCS) involved a multistage process, starting with defining measurement objectives. This was followed by a thorough literature review, phenomenological analysis, expert review, and ultimately, validation of the factor structure through Exploratory Factor Analysis (EFA). Although the findings from the EFA did not support our predictions regarding the five-factor structure, all items were still successfully retained in the new four-factor structure, namely the entertainment factor consisting of ten items, the interaction factor consisting of five items, the transaction factor consisting of three items and the recreation factor consisting of two items.

This structure explained 66.89 % of the total variance. Although researchers recommended including at least three or more items in each subscale [61], retaining the recreation subscale which had an alpha coefficient above the threshold of 0.6, namely 0.849, was chosen. These results indicated that the items on this subscale had satisfactory differentiating power [62]. Other researchers stated that subscales with fewer than three items may be retained as long as the items demonstrated a high level of internal consistency [63,64].

The article "Development and psychometric evaluation of the Employee's Workplace Cyberloafing Scale (EWCS)" was published in 2024. Journal: Heliyon.

In general, the findings from the convergent validity assessment showed that all EWCS factors and indicators can effectively capture and represent the phenomenon of cyberloafing in employees with AVE and CR values above the specified threshold. In addition, the multidimensional nature of the EWCS supported the previous scale development of [35,65], and [37].

The development of EWCS had the following scientific contributions: First, two different approaches, namely deductive and inductive, were used, while most research only used literature reviews as a deductive approach [66]. The deductive approach involved a literature review to understand the cyberloafing measurement construct and identify gaps, while the inductive approach used qualitative methods to further refine the parameters of the measurement construct. These two methods were used to complement each other in developing items from the EWCS. Second, the EWCS is an instrument that is unique in measuring cyberloafing in employees. Organizations are consistently aligning their business strategies with changing digital technologies digital (e.g., big data, IoT, AI) that present challenges for their workforce [67].

Digital transformation has led to the widespread use of digital tools in work activities, such as personal mobile devices such as tablets and smartphones [68]. In addition to increasing autonomy in the workplace [69], this evolution facilitates the emergence of new manifestations of cyberloafing such that currently existing instruments are no longer adequate to accurately assess cyberloafing. As shown in this research, the EWCS provides a comprehensive assessment of cyberloafing among employees in Indonesia. This assessment allows for a deeper understanding and interpretation of the impact of cyberloafing in the contemporary work environment. Widyastuti & Hidayat (2018) [70] stated that high employee performance is related to behavior that is relevant to organizational goals. According to Indrayanti & Ulfia, 2022 [71], elements of culture and leadership have a significant influence in fostering positive behavior in the workplace. Visionary transformative leadership and a good and healthy corporate culture, especially in implementing distributive justice in a control mechanism for all individuals in the company, can reduce the level of cyberloafing significantly [10]. Apart from that, value factors also play a role in determining employees' behavioral choices [65], whether to carry out cyberloafing or not. Good values, which were initially conditioned by a strict and effective control mechanism, were then directed towards understanding the existence of cyberloafing with positive goals such as reading news and information to enrich knowledge and improve work skills, as well as interacting online with family or friends who can create positive states of mind and emotions so that they can work more productively [11]. Moreover, if cyberloafing can later be identified with this developed instrument, then organizations also need to ensure the role of leaders, culture, and individual values in carrying out tasks.

The article "Development and psychometric evaluation of the Employee's Workplace Cyberloafing Scale (EWCS)" was published in 2024. Journal: Heliyon.

## 6 Conclusion and implication

Cyberloafing is a multifaceted phenomenon, encompassing both the “dark side” and the “light side.” This research seeks to describe the development and validation of the cyberloafing construct in current organizations. In summary, the findings of this study indicate that the EWCS has unique characteristics containing 20 items with a four-factor structure developed based on the structure and meaning of the construct determined through deductive and inductive approaches. In particular, this instrument supports the construct of cyberloafing as a multidimensional concept. The EWCS, with its high level of validity and reliability, offers researchers the opportunity to examine the antecedents, correlates, and/or consequences of cyberloafing. Finally, our findings provide significant contributions to the field of I/O psychology, especially the study of cyberpsychology.

We have presented the development of an EWCS designed to evaluate the occurrence of cyberloafing among employees. The existence of empirical findings supporting the convergent and discriminant validity of the EWCS is considered because we believe the EWCS represents one of the best options. The results of implementing EWCS include the four EWCS components including items that are practically used to provide an initial understanding of employee internet usage behavior for non-work purposes. EWCS can be used in the government or private sector to develop viable and sustainable policies related to the role of digital technology in supporting employees’ well-being and resilience, and EWCS items can be used to identify tendencies towards addictive online behavior which can cause changes in mood, procrastination, and can reduce work productivity. The government or private sector having access to such information makes it possible to create personalized intervention programs specifically to target employee mental health concerns.

## 7 Limitations and future research

This series of research has limitations that must be considered when concluding the research results. We used semi-structured in-depth interviews to gain a comprehensive understanding of the construct. However, because of the nature of individual responses which tends to be socially acceptable, the information obtained may be incomplete [66]. To gain a more comprehensive understanding, future researchers can use case study methods in various types of government organizations. A further potential limitation relates to instrument construction which is limited to the number of indicators in each component. Among the four components of EFA results, the recreation factor is the only component that has two items. Although both items demonstrated strong internal consistency, additional analysis and discussion are needed to fully understand these findings.

The article "Development and psychometric evaluation of the Employee's Workplace Cyberloafing Scale (EWCS)" was published in 2024. Journal: Heliyon.

The existing constraints indicate the need to develop instruments with many indicators so that each factor produced can consist of at least three items. Another study focuses on developing instruments using samples of employees in different work contexts, while this research only utilizes administrative employees at state universities as research samples. Sample diversification is very important for scale development to increase the generalizability of results [66]. Overall, the robustness of the research can be further improved by expanding the sample with variations in heterogeneity from public and private sector organizations.

## CRediT authorship contribution statement

**Harlina Nurtjahjanti:** Writing – original draft, Investigation, Formal analysis, Conceptualization. **Rahmat Hidayat:** Writing – review & editing, Supervision, Conceptualization. **Indrayanti Indrayanti:** Validation, Resources, Data curation.

## Data availability statement

Data will be made available on request.

## Ethical approval statement

This research obtained ethical permission from the Research Ethics Committee of the Faculty of Psychology, Gadjah Mada University, Yogyakarta, Indonesia, with approval No.6699/UN1/FPSi.1.3/SD/PT.April 01, 2022. In addition, before data collection, a prior consent form was submitted to all participants to be part of the research. In data management, information obtained from participants is stored anonymously to ensure that the data cannot be linked to any information to identify research participants.

## Funding statement

This research received no external financial or non-financial support.

## Declaration of competing interest

The authors declare that they have no known competing financial interests or personal relationships that could have appeared to influence the work reported in this paper.
